The article "A Narrative Review of the Usage of Creative Solutions to Enhance Disabled Patients' Quality of Life and Wellbeing by Occupational Therapists" was published in 2022. Journal: Occup Ther Int.

# A Narrative Review of the Usage of Creative Solutions to Enhance Disabled Patients' Quality of Life and Wellbeing by Occupational Therapists

**DOI:** 10.1155/2022/8976906

**Published:** 2022-11-05

**Authors:** Sarah Mohammed Alageel

**Affiliations:** Occupational Therapy Program, Rehabilitation Sciences Department, King Saud University, Riyadh, Saudi Arabia

## Abstract

**Introduction:**

Occupational therapists play a crucial role in the rehabilitation process, as they maximise patients' independence and participation in meaningful occupations by adopting creative solutions in their treatment plan. Recognizing the importance of creative work and incorporating it into daily activities can be a powerful technique for enhancing quality of life. As a result, OTs must comprehend the significance of using creativity on a daily basis with patients. Creativity has been implicit in occupational therapists' values and practices since the occupational therapy field's early days. In particular, OTs use meaningful activities to promote health, wellbeing, and independence, which have traditionally had a strong connection with creativity. Primarily, the OT uses practical exercise to create wellbeing and autonomy, which have had a healthy linkage with imagination. The OT has used creative exercise as a treatment technique since the beginning of the profession.

**Method:**

In this paper, a Narrative Review Checklist was used to carry out specific checks of manuscripts' structures and a careful selection of the articles which are included in the manuscript. In addition, articles referenced in review articles or guidelines were reviewed for inclusion. *Findings*. This review has shown that the primary motivation for implementing creative activities was to improve the patient performance, wellbeing, and self-esteem. The goal of implementing creative activities was to assist the client in self-expression as well as experience joy and desire. As a result, the necessity to investigate the influence of creative solutions in treatment from an OT standpoint has been identified.

**Conclusion:**

Future studies should focus on how it is important to consider the patient's intrinsic and extrinsic motivations when designing creative solutions, as well as how the disability affects their daily activities, occupations, and adherence to a treatment plan.

## 1. Introduction

The WHO defines disability as a psychological or physical deficiency affecting one's ability to perform tasks with equal competency to others of a similar age World Health Organization [WHO] [1]. Disability also affects the societal characteristics of an individual's community. Lancioni et al. [2] asserted that persons with disability face participation restrictions to leisure activities due to environmental issues. Occupational therapists (OTs) play a critical role in the therapy procedure by maximising patients' independence and involvement in eloquent works [3]. Furthermore, occupational therapy (OT) treatment is described as the art and science of assisting individuals in conducting their daily activities and is important to the theory of enhanced health and wellbeing via engagement in valued occupations [4]. Gallagher true [5] stated that health and wellbeing improve when individuals can make purposeful and meaningful choices to complete everyday actions.

The article "A Narrative Review of the Usage of Creative Solutions to Enhance Disabled Patients' Quality of Life and Wellbeing by Occupational Therapists" was published in 2022. Journal: Occup Ther Int.

In addition, according to Hong and Song (2020), the production of a unique and appropriate solution, product, or solution to an open-ended project is what creativity is all about. For nearly 50 years, the topic of creativity in OT has attracted people's curiosity [6]. Everyday creativity is considered as a capability or quality present in variable degrees in all individuals and manifests itself in all parts of daily life. Understanding the function of creativity in treatment has become a focus in the field of occupational therapy due to OTs' endorsement of this viewpoint [7].

The link of employment (human action) to the development of self-actualisation, health, and quality of life (QoL) in an individual is central to the various paradigms of occupational therapy practice (Turpin and Iwama 2011, p. 8). QoL is described as the view of people of their role in life in the sense of culture and value frameworks wherein they live and concerns their objectives, yearnings, principles, and concerns; it very well may be a wide term that impressively organizes the actual prosperity, mental condition, level of adaptability, social associations, and individual feelings Chang true [8]. QoL can be considered as an interface between the wellbeing status on the one hand and the capacity to seek after life objectives (as values to advance the physical life) on the other hand. In this way, the satisfaction of essential human needs plays a critical part within the QoL.

Although the importance of creativity in OT treatments is underappreciated by OTs, the innovativeness concept as a concept to be creative in OT therapies for impaired people is important [9]. Thus, according to Ernst and Moore [9], in order to be adopted into everyday practice, innovativeness and its components require clearer logical definitions.

The aim of this review is to address the importance of being creative in treatment as an OT in the rehabilitation setting and how applying creative solutions in the treatment will enhance the patients' QoL and wellbeing.

The article "A Narrative Review of the Usage of Creative Solutions to Enhance Disabled Patients' Quality of Life and Wellbeing by Occupational Therapists" was published in 2022. Journal: Occup Ther Int.

## 2. Methodology

### 2.1. Narrative Review Construction

The present narrative review was organized through the “Narrative Review Checklist” [10] which is proposed by the Academy of Nutrition and Dietetics. Thus, we carried out specific checks of manuscripts' structures and a careful selection of the articles which are included in the manuscript.

### 2.2. Study Selection

The search was carried out in three electronic databases, PubMed, Scopus, and Google Scholar. The search strategy included studies published from January 2015 until now. However, some included review studies contained results from high-quality studies which in some cases date before 2005. The predefined search terms were “disability” or “disabled” and “occupational therapy” or “rehabilitation” and “creativity” or “creative treatment” and “wellbeing.” For a more targeted and comprehensive search, the above words were combined with other, more specific, terms such as “quality of life” or “satisfaction.”

## 3. Discussion/Summary

### 3.1. Creativity in OT and the Development of Creativity Theories

The hypothesis is based on two key assumptions. To begin with, there is a continuum of creativity ranging from low, everyday levels of innovation to the highest degrees of creativity found in historically significant innovations, performances, scientific breakthroughs, and works of art. The second major assumption is that there are different levels of creativity in everyone's work, even within the same topic. The level of creativity a person creates at any one time is a result of the creative components functioning within and around that person at that time (Hong and Song, 2020).

Dickie [11] defined creativity as a building block to meaning as it can be a means of participation, involvement, and self-expression. Primarily, OT uses practical exercises to develop wellbeing and autonomy, which have a healthy linkage to imagination. Creativity can play an essential role in the life of the disabled. Moreover, OT has used creative exercises as a treatment technique since the founding of the profession.

In addition, creativity is an effective individual practice linked to meaning making and philosophy [12]. However, although a simple idea to comprehend, it is difficult to measure. There is no standard meaning of creativeness but rather a few designations characterised by inventiveness and exploration. Trompenaars [13] described imagination as the ability to show advancement, creativity, familiarity, and adaptability. Schmid [14] described creativity as the innate ability to act inventively and search for new and extraordinary ways of addressing issues. It has been established that creative treatments can address problems experienced by patients and greatly improve their wellbeing [14]. Moreover, OTs' creative practices have been continually proven to yield positive results with patients since the establishment of the field. It has been suggested by Maslow [15] that there are three inventiveness classes based on one's command of the necessity chain: significant imagination with connective and psychological drives, optional innovativeness with challenging and essential work, and coordinated classification which fuses the auxiliary and essential drives to attain self-actualisation. “Stream” is another imaginative hypothesis regarding the full contribution's abstract condition in any action. It is connected to drive to achieve self-actualisation and can focus on action, excellent direction feeling, stress, mindfulness deficiency, and a distorted sense of time.

The article "A Narrative Review of the Usage of Creative Solutions to Enhance Disabled Patients' Quality of Life and Wellbeing by Occupational Therapists" was published in 2022. Journal: Occup Ther Int.

OTs' primary instruments from the initial training phases in the 1960s were speciality rehearsals, and human experience expressions have been reported by a number of published studies [16]. There are a large number of published studies that describe the expressions of education and training of human artworks, and experience components have been condensed since the 1960s [17–21]. The innovativeness idea as the idea to be innovative in OT treatments for disabled patients is noteworthy, although the significance of imagination in OT treatments remains insufficiently comprehended by OTs [6, 9]. Thus, Ernst and Moore [9] suggested that innovativeness and its elements require better logical definitions to be implemented into ordinary practice.

It has been noted by Schmid [6] that OT has been enhanced by incorporating human artworks and expressions of experience into imaginative practices. The convention is entrenched in the connection between wellbeing and imagination to offer patients an opportunity to communicate their emotions and develop their learning, critical thinking, and mindfulness [22]. In his study, Schmid [6] gathered OT specialists with experience in operating creative exercises, aiming to understand the importance of inventiveness in OT. He recorded some subjects defining inventiveness as an aspect of daily living that involves critical thinking and risk-taking while other OT advisors illustrated that a positive environment is essential for such exercises to be effective. Atkinson and Wells [23] demonstrated a need to acknowledge and utilise creativity in every treatment interaction progression to ensure that OTs work effectively.

A much-debated question is whether the individual can be creative or not. Schmid [14] reported that each individual either is or has the potential to be creative. Sawyer [24] used this perspective to encourage individuals to use creativity to improve health, finding a positive effect primarily on mental recovery.

The article "A Narrative Review of the Usage of Creative Solutions to Enhance Disabled Patients' Quality of Life and Wellbeing by Occupational Therapists" was published in 2022. Journal: Occup Ther Int.

Healthcare creativity has a strong correlation with the initial therapeutic models in helping to develop healthy and stable relationships between patients and therapists [25]. While OT applies meaningful, creative activities for the promotion of independence, health, and wellbeing, Townsend [26] has reported that engaging in creative occupations is the primary human requirement that assists in organization and enhances self-efficacy, enabling individuals to manage their time effectively and manage and express their social identity.

Furthermore, creativity helps motivate individuals to continually pursue their interests [27]. It has been argued that the “just-right challenge” is a creative activity for patients to improve basic muscle movement and enhance their motivation to participate in meaningful activities as OTs play a substantial role in supporting patients' enthusiasm and engagement [22]. Additionally, creative pursuits heighten patients' self-esteem and happiness and help in resolving issues.

Finally, creativity in daily undertakings increases patients' happiness by involving them in activities aligned with their interests. According to Schmid [14], the recognition of the significance of creative work and embracing it in daily activities can be a powerful method to treat depression. OTs must understand the importance of the daily application of creativity [23].

### 3.2. Creativity in OT Practice and Theories

Although the importance of creativity in OT treatments is underappreciated by OTs, the innovativeness concept as a concept to be creative in OT therapies for impaired people is important [6, 9]. Thus, according to Ernst and Moore [9], in order to be adopted into everyday practice, innovativeness and its components require clearer logical definitions.

Patients' and OTs' beliefs significantly impact OTs' creative process. The patients' beliefs, awareness, and understanding of their disability affect OTs' initial reasoning. Shafaroodi true [28] proposed that OTs should provide patients with a description of their condition and its impacts. The extent to which a patient is aware and accepting of their condition affects their willingness to assist themselves.

Individual therapist's beliefs and values also affect OTs' creative processes. The therapist's confidence and belief in their ability to fulfil patients' needs are significant factors affecting patient-therapist interaction. In order for the creative process to be successful, OTs must have confidence in their treatment of patients Shafaroodi true [28].

The article "A Narrative Review of the Usage of Creative Solutions to Enhance Disabled Patients' Quality of Life and Wellbeing by Occupational Therapists" was published in 2022. Journal: Occup Ther Int.

Society's attitude towards disability is another aspect that impacts creative processes. There are many shortcomings of modern society affecting disabled people. Therapists should consider this when designing and prescribing assistive tools Shafaroodi true [28] as patients can easily be discouraged from active public participation. Negative attitudes towards disabled people influence patients' self-esteem and acceptance of their condition.

## 4. Conclusion

QoL and wellbeing are of great concern in OT since they affect one's ability to feel satisfaction, joy, wellbeing, solace, and balance. QoL can be considered as an interface between the wellbeing status on the one hand and the capacity to seek after life objectives (as values to advance the physical life) on the other hand.

OT should explore the role of creative occupations more deeply as an expression of intrinsic motivation and its possible use in therapeutic processes. Participating in meaningful activity is crucial to nurturing a sense of wellbeing [29].

The aim of this review was to better understand how occupational therapists use creative activities in practice in order to enhance patients' QoL and wellbeing.

Future studies should concentrate on how research can move beyond gathering demographic predictors of secondary illnesses to generating solutions that satisfy the needs of people with disability and enhance their QoL. This might be accomplished by changing the approach, methodology, and focus of rehabilitation research, for example.

People with disability complain, perhaps unsurprisingly, that they have invested time and energy in research that appears to them to be of little relevance as stated by Abma [30] or that has ended up “in a desk drawer” [30], with no apparent commitment from researchers to ensure that research findings are translated into action.

To conclude, this review suggests that it is important to consider the patient's intrinsic and extrinsic motivations when conducting future research, as well as how disability affects their daily activities, occupations, and adherence to a treatment plan. In addition, people with disability do not seek sympathy. Providing them with a creative solution for their leisure activities, on the other hand, may have a good impact on their QoL and wellbeing.

## 5. Key Findings

1. The primary motive for integrating creative activities, according to this review, was to increase patient performance, wellbeing, and self-esteem
2. The purpose of establishing creative activities was to help the client express themselves while also experiencing joy and desire
3. The need to look at the impact of creative solutions in treatment from an occupational therapy perspective has been established

The article "A Narrative Review of the Usage of Creative Solutions to Enhance Disabled Patients' Quality of Life and Wellbeing by Occupational Therapists" was published in 2022. Journal: Occup Ther Int.

## 6. What the Review Has Added

Occupational therapists should be able to produce creative ideas and solutions when treating patients with disability in the rehabilitation phase and before discharge to increase independency and therefore their quality of life and wellbeing.
